The article "ALK7 Knockdown Plays a Protective Role on HG-Stimulated MCs through Activation of the Nrf2/HO-1 Pathway" was retracted in 2023. Reasons: signs of a paper mill; compromised peer review; unreliable results or conclusions.

# ALK7 Knockdown Plays a Protective Role on HG-Stimulated MCs through Activation of the Nrf2/HO-1 Pathway

**DOI:** 10.1155/2022/4064733

**Published:** 2022-09-26

**Authors:** Shan Gao, Guifu Wu, Hui Li, Yuan Qiao, Chunping Dong

**Affiliations:** Department of Endocrinology, Shaanxi Provincial People's Hospital, Xi'an 710068, China

## Abstract

**Objective:**

Activin receptor-like kinase 7 (ALK7) is a member of the ALK family that has a key role in diabetes. However, the role of ALK7 in diabetic nephropathy (DN) remains unclear.

**Methods:**

Herein, we evaluated the effects of ALK7 on mesangial cells (MCs**).** MCs were transfected with si-ALK7 or pcDNA3.0-ALK7, and then stimulated with 40 mM glucose for 24 h. Cell proliferation was detected by MTT assay. Relative ROS level was detected using DCFH-DA staining. The contents of inflammatory cytokines were determined by ELISA. Western blot analysis was used to determine the expression levels of FN, Col IV, Nrf2, and HO-1 in MCs.

**Results:**

Our results showed that ALK7 expression was induced by HG in MCs. Knockdown of ALK7 inhibited HG-induced cell proliferation. The HG-induced ROS was mitigated by si-ALK7 with decreased ROS level and NOX activity. In addition, ALK7 knockdown exhibited anti-inflammatory activity in HG-stimulated MCs. Moreover, ALK7 knockdown attenuated fibronectin (FN) and collagen IV (Col IV) expression in MCs. Knockdown of ALK7 enhanced Nrf2/HO-1 pathway in MCs. Inhibition of Nrf2 reversed the protective effects of ALK7 knockdown on HG-stimulated MCs.

**Conclusion:**

ALK7 knockdown exerted protective effects on HG-stimulated MCs through activation of the Nrf2/HO-1 pathway. Thus, targeting ALK7 might be a therapeutic approach for the treatment of DN.

## 1. Introduction

Diabetic nephropathy (DN) is the main complication in patients with diabetes mellitus, remains a deadly chronic disease worldwide [1, 2]. Many crucial factors including dyslipidemia, poor glycemic control, smoking, and environmental and genetic clues play important roles in DN progression [1]. In recent years, many researches have uncovered the mechanisms underlying the development of DN to explore molecular targets for the treatment of DN [3–5].

During hyperglycemia, overproduction of reactive oxygen species (ROS) leads to cellular redox imbalance [6]. In addition, oxidative stress may damage mitochondrial deoxyribonucleic acid (mtDNA), therefore resulting in increased ROS production [7]. Besides, hyperglycemic state unchains an upregulation in Advanced Glycation End Products (AGEs) that induces activation of NF-*κ*B and protein kinase C (PKC) system, initiating the inflammatory response. Activation of several inflammatory cytokines, profibrotic, and vascular growth factors could promote extracellular matrix (ECM) accumulation. The microinflammation and subsequent ECM expansion are regarded as common pathways for the progression of DN [8]. Therefore, the identification of various molecules related to the oxidative stress and ECM accumulation pathways may be new therapeutic strategies for DN.

The article "ALK7 Knockdown Plays a Protective Role on HG-Stimulated MCs through Activation of the Nrf2/HO-1 Pathway" was retracted in 2023. Reasons: signs of a paper mill; compromised peer review; unreliable results or conclusions.

Activin receptor-like kinase 7 (ALK7) is a type I receptor of the transforming growth factor-beta (TGF-beta) superfamily, and mainly mediates the biological effects of GDF-1, GDF-3, Nodal, and Activin B ligands. The signaling pathway mediated by ALK7 plays an important role in cell apoptosis, proliferation, and tissue development, and is involved in neuromuscular diseases, endocrine disorders, obesity, tumors, and other diseases. ALK7-related signaling pathways have some important regulatory effects on the body [9–11]. High level of ALK7 is observed in breast cancer tissues and ALK7 overexpression inhibited cell growth and adhesion [12]. ALK7 also promoted vascular smooth muscle cells (VSMCs) phenotypic modulation [13]. In recent years, a domestic clinical study reported that the SNPrs13010956 gene polymorphism of the ALK7 gene was significantly correlated with the carotid intima-media thickness in patients with metabolic syndrome. And related animal experiments found that after the ALK7 gene was inhibited in diabetic rats, the degree of aortic sclerosis was significantly improved. [14]. ALK7 mediates H9c2 cardiomyoblast apoptosis under HG condition [15]. ALK7 gene silencing attenuated hyperlipidemia in type 2 diabetic rats [16]. Moreover, ALK7 expression is increased significantly in obstructed rat kidney [17]. However, the role of ALK7 in DN is still unclear. Herein, we evaluated the effects of ALK7 on mesangial cells (MCs).

## 2. Materials and Methods

### 2.1. Cell Culture and Treatment

Rat MC line HBZY-1 (China Center for Type Culture Collection, Wuhan, China) was cultured in RPMI-1640 medium. The HBZY-1 cells were cultured in a humidified 5% CO_2_ incubator. For the normal glucose (NG) group, cells were incubated in 5 mM glucose; for HG group, cells were incubated in 40 mM glucose.

### 2.2. Cell Transfection

The full-length ALK7 cDNA was cloned into the pcDNA3.0 plasmid (Invitrogen Corporation, San Diego, CA, USA) to construct the ALK7-overexpressing plasmid, pcDNA3.0-ALK7. The mammalian expression vector pcDNA3.0 was used as the transfection control. si-ALK7 and si-Nrf2 were obtained from RiboBio Co. Ltd.. HBZY-1 cells were transfected using lipofectamine 2000 (Invitrogen).

### 2.3. Cell Proliferation Assay

Cell proliferation was assessed by MTT method. HBZY-1 cells were seeded and incubated with MTT (0.5 mg/ml) at 37°C, and then dissolved by adding with DMSO. The absorbance (490 nm) was measured.

The article "ALK7 Knockdown Plays a Protective Role on HG-Stimulated MCs through Activation of the Nrf2/HO-1 Pathway" was retracted in 2023. Reasons: signs of a paper mill; compromised peer review; unreliable results or conclusions.

### 2.4. Measurement of ROS Detection

The cellular ROS production was analyzed using 7'-Dichlorodihydrofluorescein Diacetate (DCFH-DA) staining (Sigma-Aldrich, USA) according to the manufacturer's instruction. Briefly, about 1 × 10^4^ cells were plated on 96-well black dishes in the standard culture medium and were cultured overnight. Cells were stained with DCFH-DA (100 *μ*M), and the fluorescence intensity of different groups was analyzed by a fluorescent reader by 540 nm emission wavelength of and 480 nm excitation wavelength of.

### 2.5. NOX Activity

NOX activity was determined as previously described [18]. Briefly, homogenize tissue (10 mg) or cells (1 × 10^6^) with 200 *μ*l ice cold NADH Oxidase Lysis Buffer on ice. Centrifuge at 10000 xg and 4°C for 10 min to remove cell debris and save the supernatant. Add 1-50 *μ*l of the Sample supernatant into a 96-well white plate with flat bottom. Bring the volume of all Sample wells to 50 *μ*l with NADH Oxidase Assay Buffer. Prepare one well as Blank well in which you put 50 *μ*l of NADH Oxidase Assay Buffer. Dilute Lactate Standard to 1 mM (1 nmol/*μ*l) by adding 10 *μ*l of 100 mM Lactate Standard to 990 *μ*l dH2O, mix well. Dilute 1 mM Lactate Standard solution further to 25 *μ*M Lactate Standard (25 pmol/*μ*l) by adding 10 *μ*l of 1 mM Lactate Standard solution to 390 *μ*l of dH2O. Add 0, 2, 4, 6, 8, 10 *μ*l of 25 *μ*M Lactate Standard into a series of wells in 96-well white plate to generate 0, 50, 100, 150, 200, 250 pmol/well Lactate Standard. Adjust the volume of all Standard wells to 50 *μ*l with NADH Oxidase Assay Buffer. Add 5 *μ*l of reconstituted NADH Oxidase Positive Control into desired well(s) and adjust the volume to 50 *μ*l/well with NADH Oxidase Assay Buffer. Mix enough reagents for the number of assays to be performed. Measure the fluorescence (Ex/Em = 535/587 nm) in a kinetic mode for 30-40 min at RT. Subtract 0 Standard reading from all standard readings. Plot the Lactate Standard Curve. Subtract the Blank readings from the Sample readings. Apply the corrected Sample reading to the Lactate Standard Curve to get B pmol of Lactate generated during the reaction time (∆T = T2 − T1). The activity was valculated.

### 2.6. RT-qPCR

Total RNA extracted by TRIzol reagent was transcribed into cDNA using a PrimeScript™ RT reagent kit. This assay was performed using SYBR Green Mix. Finally, relative mRNA levels were quantified by 2^−*ΔΔ*Ct^ method.

### 2.7. Western Blot

Whole protein was extracted with cell lysis buffer. After that, 30 *μ*g protein per lane was fractionated on 10% SDS-PAGE, and then transferred onto PVDF membrane. After that, the membranes were incubated with nonfat milk. Primary antibodies against FN, Col IV, ALK7, Nrf2, lamin B2, HO-1, NQO-1, and *β*-actin (Abcam) and secondary antibody conjugated to HRP (1: 3000; Abcam) were, respectively, added to the membranes. Finally, chemiluminescent substrate was then used to visualize the bands.

The article "ALK7 Knockdown Plays a Protective Role on HG-Stimulated MCs through Activation of the Nrf2/HO-1 Pathway" was retracted in 2023. Reasons: signs of a paper mill; compromised peer review; unreliable results or conclusions.

### 2.8. ELISA

The levels of FN, Col IV, TNF-*α*, IL-1*β,* and IL-6 were analyzed by ELISA kits (eBioscience, USA) according to the manufacturer's guidance. All standards and samples were tested in the SpectraMax M5 microplate reader device at 450 nm. The standard curve was prepared, and the concentration of samples was calculated according to the absorbance value.

### 2.9. Ethical Considerations

The trial was carried out in accordance with the trial protocol and in accordance with the International Council for Harmonisation Good Clinical Practice standards. Each site's institutional review boards or independent ethics committees accepted the procedure. In accordance with the principles of the Helsinki Declaration, all patients provided written informed consent. Data on safety and efficacy were monitored by an independent data monitoring committee. No. in Ethics: NU-WU20210203.

### 2.10. Statistical Analysis

The Shapiro-Wilk test was used to evaluate the sample's normality. The exploratory analyses of the Tukey test were used to analyze descriptive statistical data. To examine the inferential statistics, quantitative mean data (PES/WES, ISQ, and B.L.) were tested using the nonparametric Wilcoxon-Mann–Whitney *U*-test. Experimental data are presented as mean ± S.D. ANOVA was performed to show the difference between groups. *p* < 0.05 was considered as significant difference.

## 3. Results

### 3.1. ALK7 Expression Was Increased in HG-Stimulated HBZY-1 Cells

We first examined whether ALK7 expression could be regulated by HG stimulation. The results of Figure 1(a) showed that ALK7 mRNA level was markedly increased by HG. Similarly, HG stimulation also significantly upregulated ALK7 protein expression in HBZY-1 cells (Figure 1(b)).

### 3.2. Knockdown of ALK7 Inhibited MC Proliferation

To investigate the role of ALK7 in HBZY-1 cells, si-ALK7 was transfected into the cells. ALK7 protein expression in HBZY-1 cells was significantly reduced following transfection with si-ALK7, as seen in Figure 2(a). In addition, HG could promote cell proliferation; while the increased MCs proliferation was deceased in si-ALK7 transfected HBZY-1 cells (Figure 2(b)).

### 3.3. si-ALK7 Inhibited HG-Induced ROS Level in HBZY-1 Cells

We measured the effect of si-ALK7 on ROS level and NOX activity. The ROS level showed a significant increase in the HG-stimulated HBZY-1 cells, which was reduced by si-ALK7 (Figures 3(a) and 3(b)). Next, the NOX activity was determined and NOX activity was upregulated in HBZY-1 cells under HG, while the effect was reversed by knockdown of ALK7 (Figure 3(c)).

The article "ALK7 Knockdown Plays a Protective Role on HG-Stimulated MCs through Activation of the Nrf2/HO-1 Pathway" was retracted in 2023. Reasons: signs of a paper mill; compromised peer review; unreliable results or conclusions.

### 3.4. si-ALK7 Inhibited Proinflammatory Cytokines in Cells

The levels of inflammatory cytokines were measured by RT-qPCR and ELISA. As indicated in Figures 4(a)–4(c), increased TNF-*α*, IL-1*β*, and IL-6 mRNA levels in HG-stimulated HBZY-1 cells were decreased by si-ALK7. The upregulated levels of these cytokines in supernatant of HG-stimulated HBZY-1 cells were also suppressed by knockdown of ALK7 (Figures 4(d)–4(f)).

### 3.5. Knockdown of ALK7 Repressed ECM Production in HBZY-1 Cells

ECM accumulation plays critical roles in DN progression. Next, we examined the effects of ALK7 on ECM proteins in cells. The results from ELISA proved that production was significantly higher in HG-stimulated HBZY-1 cells. However, knockdown of ALK7 significantly repressed HG-increased FN and Col IV production (Figures 5(a) and 5(b)). In addition, we observed HG-induced two proteins expression was also reversed by ALK7 knockdown in HG-stimulated HBZY-1 cells (Figures 5(c) and 5(d)).

### 3.6. ALK7 Promoted Inflammation and ECM in HBZY-1 Cells

In addition, cells were transfected with ALK7-overexpressing plasmid to confirm the role of ALK7.  Figure 6(a) shows that LK7 protein level was increased by pcDNA3.0-ALK7 in the HG-stimulated HBZY-1 cells. In addition, the elevated cell proliferation and ROS level in HG-treated HBZY-1 cells were enhanced by ALK7 overexpression (Figures 6(b) and 6(c)). Moreover, HG-induced productions of inflammatory cytokines were aggravated by ALK7 overexpression (Figures 6(d)–6(f)). Furthermore, the HG-caused increases in ECM protein expression were also enhanced in ALK7-overexpressing HBZY-1 cells (Figures 6(g) and 6(h)).

### 3.7. si-ALK7 Enhanced Nrf2/HO-1 Pathway in HBZY-1 Cells

We examined the effect of si-ALK7 on this pathway. HG stimulation slight increased Nrf2 and HO-1 expression. However, these effects were significantly enhanced by knockdown of ALK7 (Figures 7(a)–7(c)).

### 3.8. Si-ALK7 Increased NQO-1 Level in HBZY-1 Cells

Subsequently, the effect of si-ALK7 on expression level of Nrf2-driven gene, such as NQO-1 was assessed. The protein level of NQO-1 was increased by HG, and the effect was greatly enhanced by si-ALK7 (Figures 8(a) and 8(b)).

### 3.9. Si-Nrf2 Reversed Protective Effects of ALK7 Knockdown on HBZY-1 Cells

Finally, HBZY-1 cells were transfected with si-Nrf2. si-Nrf2 reduced nuclear expression of Nrf2 transfected with si-ALK7 following HG (Figures 9(a) and 9(b)). In addition, the ALK7 knockdown-caused decreases in production of ROS, TNF-*α*, IL-1*β*, and IL-6 were upregulated after transfection with si-Nrf2 (Figures 9(c)–9(f)). Furthermore, the effects of si-ALK7 on FN and Col IV production were reversed by si-Nrf2 (Figures 9(g) and 9(h)).

The article "ALK7 Knockdown Plays a Protective Role on HG-Stimulated MCs through Activation of the Nrf2/HO-1 Pathway" was retracted in 2023. Reasons: signs of a paper mill; compromised peer review; unreliable results or conclusions.

## 4. Discussion

ALK7 can participate in the regulation of cell proliferation, differentiation, apoptosis, and adhesion through non-Smads signaling pathway molecules. The expression of ALK7 is found in various tissues and cells, and it is relatively specific for adipose tissue. In recent years, a large number of studies have found that ALK7 plays a role in maintaining metabolic homeostasis in the body. Under the action of ligand nodal and other proapoptotic signals, ALK7 is upregulated and then activates downstream signaling pathways such as Smad, which can promote the apoptosis of islet *β* cells, and can inhibit the stimulating effect of high glucose on the release of insulin from *β* cells, resulting in increased blood sugar. Similarly, in adipose tissue metabolism, AKL7 can participate in the differentiation of adipocytes by mediating the growth differentiation factor 3 (GDF3) signaling pathway, causing the accumulation of adipose tissue in the body, aggravating insulin resistance, and leading to the occurrence of obesity; hyperglycemia can also upregulate ALK7 expression, which in turn acts on the pancreas to reduce insulin release and insulin resistance, resulting in a vicious circle of continuous rise in blood sugar. Herein, our results demonstrated that HG-induced upregulated ALK7 expression in HBZY-1 cells. ALK7 regulated proliferation and ECM accumulation in HG-stimulated HBZY-1 cells.

TGF-*β* superfamily includes TGF-*β*s, Nodal, Inhibins, BMPs, and GDFs [19, 20]. TGF-*β* family members regulate cell proliferation, apoptosis, and differentiation [21]. ALKs (include seven members ALK1-7) is type I receptor of TGF-*β* family and expressed in pancreatic islets and *β*-cell lines [22]. It has been shown that pancreatic islets show different gene-expression profiles of ALK7 at various glucose concentrations, indicating that the extracellular glucose condition regulates the expression of the genes of activins and ALKs [23, 24]. In this study, we discovered that HG increased ALK7 expression in HBZY-1 cells. In HG-stimulated cells, si-ALK7 decreased inflammation and ECM buildup, but ALK7 overexpression had the opposite effect, showing that ALK7 may regulate the course of DN. Previous research found that ALK7 knockdown protects osteoblast cells from high glucose-induced ROS generation via Nrf2/HO-1 signaling [25]. The silencing of ALK7 represses high glucose-induced apoptosis and oxidative stress in retinal pigment epithelial cells ([14] #2). Our finding is consistent with the previous studies and enriches the understanding of the function of ALK7.

The article "ALK7 Knockdown Plays a Protective Role on HG-Stimulated MCs through Activation of the Nrf2/HO-1 Pathway" was retracted in 2023. Reasons: signs of a paper mill; compromised peer review; unreliable results or conclusions.

Nrf2 is a redox-sensitive transcription factor [26]. Under stimulus, the sequestered Nrf2 regulates some antioxidant enzymes expression via ARE [26, 27]. Nrf2/HO-1 pathway is involved DN progression. Nrf2/HO-1 attenuates HG-induced EMT in renal tubule cells [28]. Activation of Nrf2/HO-1 prevents ROS development, and inhibits apoptosis in renal tubule cells [29]. Chlorogenic acid prevents DN progression by repressing inflammation and oxidative stress via Nrf2/HO-1 pathway [30]. Sinapic acid ameliorates streptozotocin-induced DN in rats through its anti-inflammatory and antioxidative effects via Nrf2/HO-1 mediated pathways [31]. In addition, ALK7 knockdown protected ARPE-19 cells against HG-induced injury via Nrf2/HO-1 pathway [14]. Our results proved that si-ALK7 enhanced Nrf2/HO-1 pathway in HBZY-1 cells. And, inhibition of this pathway reversed the effects of ALK7 knockdown on HBZY-1 cells.

For DN, the research on its mechanism for a long time has mainly focused on the changes of blood components directly acting on the process of kidney injury; however, diabetes is not only a change in blood components but a chronic inflammatory disease affecting multiple systems in the body. Among them, in the early stage of diabetes, due to the increased release of proinflammatory factors and the down-regulated secretion of anti-inflammatory factors, a series of pathological changes can occur in the adventitia of blood vessels rich in fibroblasts. However, so far, its specific mechanism is not fully understood and needs to be further explored. Our findings provide a certain reference value for the future precision treatment of DN and early clinical diagnosis and screening. By understanding the elevated level of DN blood glucose, it is possible to predict the upregulation of ALK7 expression in vivo, which may also be a direction for future drug design. There are still some limitations in the current work. For example, the fluorescent probe DCFH-DA is used to determine “ROS production”, but the probe may be not specific, especially in complex biological samples such as the ones used in the present work [32], and other more specific method should be performed in the future investigations [33].

In conclusion, the expression of ALK7 was found in rat MCS cells for the first time; the knockdown exerted protective effect of ALK7 on MCs through Nrf2/HO-1 pathway was clarified; it was verified that ALK7 was involved in the phenotype transformation of Rat MC line HBZY-1 and the increase in collagen synthesis. Therefore, targeting ALK7 might be a therapeutic approach DN. It provides some ideas for the determination of new epigenetic targets for the clinical diagnosis and prognosis of DN in the future. However, given the limitations of this study, future protein model construction and drug design need to be further studied.

The article "ALK7 Knockdown Plays a Protective Role on HG-Stimulated MCs through Activation of the Nrf2/HO-1 Pathway" was retracted in 2023. Reasons: signs of a paper mill; compromised peer review; unreliable results or conclusions.

## Figures and Tables

**Figure 1:** HG induces ALK7 expression in MCs. (a) The mRNA expression pattern of ALK7 in MCs was examined by RT-qPCR in response to 40 mM glucose stimulation for 24 h. (b) The protein expression pattern of ALK7 in MCs was examined by western blot after stimulation with 40 mM glucose for 24 h. ^∗^*p* < 0.05 vs. NG group.

**Figure 2:** Knockdown of ALK7 inhibits MCs proliferation in HG-stimulated MCs. (a) Relative protein expression levels of ALK7 were detected by western blot after transfection with si-ALK7 or si-con in HG-stimulated MCs. (b) MTT assay was used to detect cell proliferation. ^∗^*p* < 0.05 vs. NG group. ^#^*p* < 0.05 vs. HG + si − NC group.

**Figure 3:** Knockdown of ALK7 inhibits ROS level and NOX activity in HG-stimulated MCs. (a and b) Relative ROS levels with different treatments. (c) NADPH oxidase activity in MCs with different treatments. ^∗^*p* < 0.05 vs. NG group. ^#^*p* < 0.05 vs. HG + si − NC group.

**Figure 4:** Knockdown of ALK7 inhibits the production of TNF-*α*, IL-1*β*, and IL-6 in HG-stimulated MCs. (a–c) The mRNA levels of TNF-*α*, IL-1*β*, and IL-6 in MCs were measured by RT-qPCR. (d–f) The contents of TNF-*α*, IL-1*β*, and IL-6 were determined by ELISA. ^∗^*p* < 0.05 vs. NG group. ^#^*p* < 0.05 vs. HG + si − NC group.

**Figure 5:** Knockdown of ALK7 attenuates FN and Col IV production in HG-stimulated MCs. (a and b) The contents of FN and Col IV in supernatant of MCs were determined by ELISA. (c and d) FN and Col IV protein expressions were measured by western blot. ^∗^*p* < 0.05 vs. NG group. ^#^*p* < 0.05 vs. HG + si − NC group.

**Figure 6:** ALK7 enhances HG-induced production of ROS, inflammatory cytokines and ECM proteins in MCs. (a) ALK7 protein expression was detected by western blot after transfection with pcDNA3.0-ALK7 in HG-simulated MCs. (b) Cell proliferation was detected. (c) Relative ROS levels in MCs with different treatments. (d–f) The contents of inflammatory cytokines were determined by ELISA. (g and h) The protein levels of FN and Col IV in MCs were measured by western blot. ^∗^*p* < 0.05 vs. NG group. ^#^*p* < 0.05 vs. HG + pcDNA3.0 group.

**Figure 7:** Knockdown of ALK7 enhances the Nrf2/HO-1 pathway in MCs. (a–c) Western blot analysis was used to determine the expression levels of Nrf2 and HO-1 in MCs. ^∗^*p* < 0.05 vs. NG group. ^#^*p* < 0.05 vs. HG + si − NC group.

The article "ALK7 Knockdown Plays a Protective Role on HG-Stimulated MCs through Activation of the Nrf2/HO-1 Pathway" was retracted in 2023. Reasons: signs of a paper mill; compromised peer review; unreliable results or conclusions.

**Figure 8:** Knockdown of ALK7 increases the expression level of NQO-1 in HG-treated MCs. (a) The protein level of NQO-1 in MCs was detected by western blot. (b) Quantification analysis of NQO-1. ^∗^*p* < 0.05 vs. NG group. ^#^*p* < 0.05 vs. HG + si − NC group.

**Figure 9:** Knockdown of Nrf2 reverses the effects of ALK7 knockdown on oxidative stress, inflammation and ECM accumulation in MCs. (a and b) Relative expression levels of Nrf2 in MCs were detected by western blot after transfection with si-Nrf2. (c) Relative ROS levels in MCs with different treatments. (d–f) The contents of inflammatory cytokines were determined by ELISA. (g and h) The contents of FN and Col IV were determined using ELISA. ^∗^*p* < 0.05 vs. NG group. ^#^*p* < 0.05 vs. HG + si − NC group. ^&^*p* < 0.05 vs. HG + si − ALK7 group.

## Data Availability

The datasets used during the present study are available from the corresponding author upon reasonable request.
